# SIRT1 Attenuates Apoptosis of Nucleus Pulposus Cells by Targeting Interactions between LC3B and Fas under High-Magnitude Compression

**DOI:** 10.1155/2021/2420969

**Published:** 2021-12-27

**Authors:** Yunyun Zhuo, Haoming Wang, Luetao Zou, Yiyang Wang, Yanzhu Hu, Pei Li, Qiang Zhou

**Affiliations:** ^1^Department of Orthopedics, The Third Affiliated Hospital of Chongqing Medical University, Chongqing 400010, China; ^2^Department of Orthopedics, Three Gorges Central Hospital, Chongqing 404000, China; ^3^Tissue Repairing and Biotechnology Research Center, The Third Affiliated Hospital of Chongqing Medical University, Chongqing 401120, China

## Abstract

Mechanical overloading-induced nucleus pulposus cell (NPC) apoptosis plays a core role in the pathogenesis of intervertebral disc degeneration. In this study, we investigated the involvement of mammalian silent information regulator 2 homolog (SIRT1) in NPC apoptosis under high-magnitude compression. Our results showed that high-magnitude compression aggravated cellular apoptosis and attenuated the expression levels of SIRT1 and microtubule-associated protein-1 light chain-3B (LC3B) in rat NPCs in a three-dimensional (3D) cell culture model and an in vivo rat tail compression model, whereas SIRT1 overexpression in NPCs partially reversed these indicators. Moreover, SIRT1 overexpression increased the formation of the LC3B/Fas complex, alleviated activation of the NF-*κ*B pathway, and reduced NPC apoptosis. Finally, downregulation of LC3B partially activated the NF-*κ*B pathway and aggravated NPC apoptosis. Overall, upregulation of SIRT1 increases formation of the LC3B/Fas complex, which contributes to suppression of NPC apoptosis by inhibiting the NF-*κ*B pathway under high compressive stress.

## 1. Introduction

Intervertebral disc degeneration (IDD) is one of the main pathological causes of low back pain worldwide, which seriously reduces the quality of life of patients and brings a heavy socioeconomic burden [1]. Intervertebral discs (IVDs) are heterogeneous structures with two facet joints that function as a “three-joint complex” to resist different mechanical loads and deformations in daily life movements, such as walking, bending, and leaning back [2]. As an important part of IVDs, the central nucleus pulposus can absorb and transmit oscillations of external forces, balance stress, and provide load support and flexibility of the spine [3, 4]. It has been widely reported that high-magnitude compression can promote apoptosis and dyshomeostasis of the extracellular matrix (ECM) of NPCs and thereby accelerate the process of IDD [2, 5, 6].

Autophagy, characterized by autophagosome formation, is an evolutionarily conserved process through which the deleterious organelles and proteins induced by cellular stress can be eliminated [7, 8]. Various chemical or physical factors, such as excessive load, nutrition deprivation, inflammation, hypoxia, and accumulation of reactive oxygen species (ROS), can induce cell autophagy [7, 9, 10]. Previous studies have shown that autophagy plays a protective role in IDD, and modulating autophagy might be an efficacious treatment for compression-induced IDD [11–13]. Conversion of microtubule-associated protein-1 light chain-3B (LC3B) from its cleaved form (LC3B-I) to LC3B-II (phosphatidyl-ethanolamine conjugated form) and the accumulation of LC3B are widely regarded as autophagy markers [11, 14]. Previous studies have reported that autophagy interacts with apoptosis via an interaction between LC3B and FAS [15, 16]. Yeganeh et al. demonstrated that stretch/ceramide-induced autophagy in rat lung epithelial cells may activate the Fas/FasL-mediated extrinsic apoptotic pathway via an LC3B and FAS interaction [17]. However, evidence of crosstalk between autophagy and apoptosis in NPCs under compressive stress is very limited.

Mammalian silent information regulator 2 homolog SIRT1 is an NAD-dependent class 3 histone deacetylase that plays a major role in the regulation of various cellular processes related to oxidative stress, metabolism, cell senescence, apoptosis, and autophagy [18–20]. Previous studies have proclaimed that SIRT1 can impede NPC apoptosis by stimulating autophagy and thereby ease the process of IDD [12, 21, 22]. Similarly, our recent study revealed that SIRT1 can attenuate high compressive stress-induced NPC senescence via PINK1-dependent mitophagy [23]. However, whether SIRT1 is involved in NPC apoptosis and autophagy under compressive stress is unclear.

Therefore, this study was performed to investigate the biological role of SIRT1 in cell apoptosis and autophagy in rat NPCs under high compressive stress and to identify whether the interactions between LC3B and Fas participate in this process.

## 2. Materials and Methods

### 2.1. Human NP Tissue Collection

NP tissues from 5 lumbar vertebral fracture (LVF) patients (3 males, 2 females; Pfirrmann I-II) and 10 IDD patients (6 males, 4 females; Pfirrmann IV-V) were acquired from the Department of Orthopedics, the Third Affiliated Hospital of Chongqing Medical University. The degeneration grades of IVD were defined according to the Pfirrmann classification system using preoperative MRI scans [24]. The procurement and use of human-derived tissue in this study were approved by the ethics committee of Chongqing Medical University.

### 2.2. Rat NPC Isolation and Scaffold Preculture

Twenty-five healthy Sprague–Dawley rats (male, 250 g, 6–8 weeks old) were obtained from the Animal Center of Chongqing Medical University. After animals were sacrificed with excessive carbon dioxide (CO_2_), the lumbar discs (L1-L5) were removed, and the innermost NP tissues were removed using a No. 11 surgical blade. Then, the NP tissues were digested with type II collagenase (0.2%, Sigma, USA) for 1-2 h, followed by trypsin solution (0.25%, Sigma, USA) for 30 min. NPC pellets were collected by centrifugation (1000 rpm for 10 min) and resuspended in complete culture medium (DMEM/F-12) (Gibco, USA) containing 10% fetal bovine serum (Gibco, USA) and 1% penicillin/streptomycin (Sigma, USA) under standard conditions (37°C, 20% O_2_, and 5% CO_2_). The cell-seeding procedure in this study was performed as described in a previous study [24]. Briefly, passage 2 NPCs at a density of 1 × 10^7^ cells/mL were premixed with liquid hydrogels (Gel-MA), which were freely provided by the Tissue Engineering Center of the Third Military Medical University. Then, the mixture was transferred into a cylindrical mold (*Ø* = 5 mm, height = 5 mm) and exposed to ultraviolet light (365 nm) for approximately 1-2 min to establish the 3D network. Then, the NPC hydrogels were precultured under standard conditions (37°C, 20% O_2_, and 5% CO_2_) for 2 days.

### 2.3. Mechanical Compression Application

The main units of the self-developed substance exchanger-based perfusion bioreactor are illustrated in Figure 1(a). The NPC hydrogels were perfusion-cultured in the bioreactor at 37°C for 5 days and simultaneously compressed at 0% (control group) or 20% (high-compression group) compressive deformation at a frequency of 1.0 Hz for 4 h once per day. After moderate digestion with type II collagenase, the NPCs in the hydrogels were harvested for subsequent experiments.

### 2.4. NPC Transfection

A recombinant lentiviral vector for SIRT1 overexpression (LV-SIRT1) and siRNA targeting LC3B (LC3B-siRNA) were obtained from GeneChem (Shanghai, China). For transfections, NPCs were seeded into 24-well plates (2 × 10^4^ cells per well). After incubation for 24 h, the cells were transfected according to the manufacturer's instructions. The transfection efficacy was verified via real-time polymerase chain reaction (PCR) and western blotting.

### 2.5. Flow Cytometry

After NPCs were washed twice with phosphate-buffered saline (PBS), cell apoptosis was analyzed via flow cytometry using an Annexin V/PI apoptosis detection kit (LIANKE, Hangzhou, China) according to the manufacturer's instructions.

### 2.6. Real-Time PCR

Total RNA was extracted using TRIzol reagent (TaKaRa) and transcribed into cDNA using a cDNA synthesis kit (Takara). Quantitative real-time PCR was conducted using a 7500 Fast Real-Time PCR System with SYBR ®Premix EX Taq™ II (TaKara). The forward and reverse primer sequences used to amplify marker genes are listed in Table 1. Reactions were performed under thermal cycling conditions of 10 sec at 95°C, followed by 40 cycles of 30 sec at 95°C and 34 sec at 60°C. *β*-Actin was used as an internal control. Relative mRNA levels were calculated using the 2^-*ΔΔ*CT^ method.

### 2.7. Western Blotting

Protein was extracted using radioimmunoprecipitation assay buffer supplemented with 1 mM phenylmethylsulfonyl fluoride (Sigma, St. Louis, MO). After the protein concentration was measured with a bicinchoninic acid (BCA) protein assay kit (Beyotime, China), the proteins were separated in 10% or 12% (*w*/*v*) sodium dodecyl sulfate polyacrylamide gels and then transferred to a 0.22 *μ*m pore size PVDF membrane (Merck Millipore). After blocked with TBST containing 5% (*w*/*v*) bovine serum albumin, the membranes were incubated with primary antibodies (anti-SIRT1: diluted at 1 : 1000, Cell Signaling Technology, USA; anti-LC3B, anti-P62, and anti-cleaved-caspase 3: diluted at 1 : 1000, Abcam, USA; anti-Bax, anti-Bcl-2, anti-P65/NF-*κ*B, anti-p-P65/p-NF-*κ*B, and anti-*β*-actin: diluted at 1 : 000, Proteintech, China) overnight at 4°C. The membranes were washed three times with cold TBST for 15 min and then incubated with horseradish peroxidase-labeled secondary antibody (Beyotime, Wuhan, China) at room temperature for 1 h. Finally, protein blots were detected via chemiluminescence (ECL-Kit, Bio–Rad, Cambridge, MA, USA) and quantified using Quantity One analysis software, version 4.4 (Bio–Rad).

### 2.8. Immunoprecipitation Assays

Cell precipitates were collected, binding buffer containing protease inhibitors was added, and the cells were lysed on ice for 1 hour. The supernatant was centrifuged at 14000 g for 15 minutes, and the protein concentration was measured. The same amount of protein sample and mouse anti-Fas antibody (diluted at 1 : 50; Santa Cruz, USA) were inverted and stirred at 4°C for 24 hours. Pretreated Protein A/G magnetic beads (Bimake, Houston, TX, USA) were added and incubated with the samples at 4°C by stirring upside down for 1 hour. The washing buffer was fully removed, and the supernatant was removed. Then, SDS loading sample buffer was added, and the samples were boiled for 10 minutes at 100°C. Subsequent western blotting was performed with 40-60 *μ*l samples added to each well according to the standard experimental steps.

### 2.9. Immunofluorescence Staining

Cells were cultured on glass coverslips, fixed with 4% paraformaldehyde and permeabilized with 0.5% Triton X-100 in PBS for 10 min at room temperature. Subsequently, nonspecific binding was blocked with 5% BSA for 1 h at room temperature, and then, the cells were incubated overnight with primary antibodies (anti-SIRT1: diluted at 1 : 1000; anti-SQSTM1/P62: diluted at 1 : 1000, Abcam, USA) at 4°C. The coverslips were washed with PBS and incubated with a Cy3 secondary antibody (diluted at 1 : 50, Proteintech, China) for1 h at room temperature. Finally, the coverslips were washed with PBS, and nuclei were stained with 4,6-diamidino-2-phenylindole (DAPI). Finally, the stained NPCs were visualized using a confocal laser scanning microscope (Leica).

### 2.10. Transmission Electron Microscopy (TEM)

The NPC hydrogels were digested with type II collagenase and then centrifuged at 1000 rpm for 15 min. The cell pellet was harvested and fixed with 2.5% glutaraldehyde overnight at room temperature. Then, NP samples were dehydrated in an ascending ethanol series and embedded in Epon 812. The samples were cut into ultrathin sections, stained with lead citrate, and finally observed using a Hitachi-7500 transmission electron microscope (Hitachi, Japan).

### 2.11. Rat Tail Compression Model

Adult Sprague–Dawley rats (female, 500 ± 5 g, 12 months old) were purchased from the Experimental Animal Center of Chongqing Medical University and randomly divided into four groups: sham group, IDD group, lenti NC group, and lenti SIRT1 group. The modified rat tail static compression model was designed as described in a previous study [25]. After successful anesthesia, under the guidance of a C-arm, an equal-length Kirschner wire with a diameter of 1.5 mm was implanted in the center of the 7th and 8th caudal vertebrae, perpendicular to the sagittal direction of the caudal vertebrae. The two Kirschner wires were always parallel to each other in the coronal position, and the distance between the Kirschner wires was measured before applying compressive deformation. Except for the sham operation group, the other three groups were subjected to 10% compressive deformation by fixing the Kirschner wire with a self-developed compression loading apparatus. According to the microinjection method reported in a previous study [26], the lenti NC or lenti SIRT1 construct was injected into the rat tail intervertebral disc. A magnetic resonance imaging (MRI) examination was performed 4 weeks later, and the target intervertebral disc was removed for subsequent HE and immunohistochemical staining.

### 2.12. HE Staining and Immunohistochemistry

After human disc NP tissues were fixed with 4% paraformaldehyde, they were embedded in paraffin and cut into slices. For the fixed intact rat discs using 4% paraformaldehyde, they were decalcified using commercial EDTA Decalcification Solution (Servicebio, G1105-500ML, China) for 2 weeks at room temperature before embedding and cutting. After being dewaxed, the slices were used for HE staining according to the standard process. Finally, the histological scores were calculated to evaluate IDD according to a histologic scoring system described by a previous study [27]. For immunohistochemistry, the tissue slices were treated with 3% H_2_O_2_ at room temperature for 10 min and blocked with 1% BSA at 37°C for 30 min. The samples were then incubated with primary antibodies (anti-LC3B, anti-cleaved caspase 3, and anti-p-P65: diluted at 1 : 100) overnight at 4°C and then with HRP-labeled secondary antibodies, followed by staining with DAB and counterstaining with hematoxylin.

### 2.13. Statistical Analysis

Statistical analyses were performed using SPSS Statistics for Windows (Version 20.0. Chicago, IL: SPSS Inc.). Differences between experimental groups were evaluated using a two-sided unpaired Student's *t*-test or one-way analysis of variance (ANOVA). Differences with a *P* value < 0.05 were accepted as statistically significant. All results represent the mean value from at least three independent experiments.

## 3. Results

### 3.1. Observation of SIRT1 Expression, Cell Apoptosis, and Autophagy in Human Degenerated NP Tissues

First, SIRT1 expression was confirmed to be associated with cell apoptosis and autophagy in human NP tissues. As shown in Figures 2(a) and 2(b), immunohistochemical results indicated that SIRT1 and LC3B expression was obviously lower in IDD tissues than in LVF tissues, whereas the expression of cleaved caspase 3 (apoptosis-related biomarker) in IDD tissues was significantly higher than that in LVF tissues. Furthermore, western blotting also demonstrated the same results: SIRT1 and LC3B expression decreased, but cleaved caspase 3 expression increased in the IDD group (Figure 2(c)). All of these data suggest that SIRT1 and LC3B expression was decreased but cell apoptosis was enhanced during IDD.

### 3.2. High-Magnitude Compression Aggravated Cell Apoptosis and Attenuated SIRT1 Expression in Rat NPCs

To further study the relationship between apoptosis and SIRT1 expression, a 3D culture model was established with rat NPCs using Gel-MA hydrogel scaffolds and a self-developed perfusion bioreactor (Figure 1(a)). The expression of SIRT1 and cellular apoptosis markers was detected after applying diverse dynamic compressive stresses (0% and 20% compressive deformation). As shown in Figure 1(b), flow cytometry analysis revealed that the apoptotic rate in the high-compression group was significantly higher than that in the control group. Furthermore, evaluation of the levels of apoptosis-related biomarkers via western blotting showed that Bcl-2 was decreased while Bax and cleaved caspase 3 were sharply increased in NPCs subjected to high compressive stress. Furthermore, the NF-*κ*B pathway was significantly activated under high-magnitude compression, indicated by the level of p-P65 protein expression (Figure 1(c)). In line with the results of western blotting (Figure 1(c)), immunofluorescence data revealed that high compressive stress reduced the expression of SIRT1 in NPCs (Figure 1(d)).

### 3.3. SIRT1 Overexpression Enhanced Autophagy and Reduced Cell Apoptosis in Rat NPCs under High-Magnitude Compression

Previous reports have shown that SIRT1 impedes apoptosis by promoting autophagy [12, 22, 28]. Hence, SIRT1 was overexpressed in NPCs using a lentiviral SIRT1 expression vector (LV-SIRT), and the status of autophagy and apoptosis in NPCs exposed to high compressive stress was examined. The efficiency of SIRT1 overexpression was confirmed via real-time PCR and western blotting (Figure 3(a)). As shown in Figure 3(b), western blotting analysis revealed that overexpression of SIRT1 under high-magnitude compression strongly upregulated the expression of LC3II/*β*-actin and Bcl-2 but downregulated the expression of P62, Bax, and cleaved caspase 3. Immunofluorescence assays and TEM analysis demonstrated that overexpression of SIRT1 increased autophagosome formation under high-magnitude compression (Figures 3(c) and 3(d)). TUNEL staining results showed that the number of TUNEL-positive cells was significantly decreased in the 20%+SIRT1 group (Figure 3(f)), which was consistent with the results of the flow cytometry analysis (Figure 3(e)).

Overall, these data suggest that high compressive stress depressed autophagy but promoted apoptosis in NPCs, while upregulation of SIRT1 partially rescued these effects.

### 3.4. SIRT1 Overexpression Increased Formation of the LC3B/Fas Complex and Inhibited Activation of the NF-*κ*B Pathway

Next, to gain insight into the mechanism by which SIRT1 overexpression can retrieve autophagy and depress cell apoptosis, immunoprecipitation was performed to examine whether LC3B interacts with FAS. As expected, SIRT1 overexpression obviously increased the formation of the LC3B/Fas complex (Figure 4(a)). NF-*κ*B signaling pathway plays a key role in IDD [29, 30]. Western blotting analysis showed that high compressive stress dramatically promoted the level of p-P65 compared to the level in the control group, whereas SIRT1 overexpression in NPCs partially reduced the p-P65 level (Figure 4(b)).

### 3.5. Downregulation of LC3B Alleviated the Inhibition of the NF-*κ*B Signaling Pathway and Aggravated Apoptosis in SIRT1-Overexpressing NPCs under High-Magnitude Compression

To further verify whether SIRT1 safeguards against compression-induced apoptosis of NPCs by prompting formation of the LC3B/Fas complex, we transfected NPCs exhibiting SIRT1 overexpression with siRNA targeting LC3B. Then, these cells were exposed to high compressive stress. As shown in Figure 5(a), the effectiveness of siRNA treatment was identified by western blotting. Next, the level of cleaved caspase 3 was analyzed using western blotting, and the result showed that the expression level of cleaved caspase 3 increased in the 20%+SIRT1+siLC3B group (Figure 5(b)) compared with that in the 20%+SIRT1 group. Additionally, flow cytometry analysis revealed that the apoptotic rate in the 20%+SIRT1+siLC3B group was significantly higher than that in the 20%+SIRT1 group (Figure 5(c)). Consistently, TUNEL staining results showed that the number of TUNEL-positive cells was significantly increased in the 20%+SIRT1+siLC3B group compared to the 20%+SIRT1 group (Figure 5(d)). Moreover, western blotting revealed that the expression level of p-P65 in the 20%+SIRT1+siLC3B group was sharply higher than that in the 20%+SIRT1 group (Figure 5(b)). These results suggest that downregulation of LC3B partially activated the NF-*κ*B signaling pathway, which may give rise to apoptosis of NPCs under high-magnitude compression.

### 3.6. SIRT1 Overexpression Rescued Autophagy and Reduced Cell Apoptosis in a Rat Tail Compression Model

Finally, a rat tail compression model was constructed to ascertain the therapeutic effect of SIRT1 in vivo (Figure 6(a)). Representative MRI scans of rat coccygeal vertebrae are shown in Figure 6(b), and the outcomes revealed a higher T2-weighted disc signal intensity in the lenti-SIRT1 transfection group (IDD+SIRT1 group) than that in the IDD or IDD+NC group. However, the IDD+NC group and IDD+SIRT1 group showed the presence of relatively high MRI signals in the vertebral bone and endplates; we deduce that there may exist some injury, inflammation, or local infection. Moreover, the IDD+SIRT1 group showed a well-organized tissue structure and extracellular matrix (ECM) distribution, whereas the severely degenerated NP tissues in the IDD group and IDD+NC group showed a lower cell density and an abnormal ECM distribution in the results of HE staining (Figure 6(c)). In line with the HE images, the IDD+SIRT1 group showed a lower histological score compared with the IDD group and IDD+NC group. Finally, the IDD+SIRT1 group showed higher LC3B protein expression and lower p-P65 and cleaved caspase 3 protein expression than the IDD group or IDD+NC group (Figure 6(d)). Collectively, these in vivo results suggest that SIRT1 may alleviate NPC apoptosis by regulating autophagy and the NF-*κ*B pathway under mechanical loading.

## 4. Discussion

It is well known that excessive or inappropriate mechanical loading is considered a crucial contributor to the development of IDD [31, 32]. Many studies have demonstrated that high compressive stress may accelerate NPC apoptosis and aggravate IDD in vitro and in vivo [2, 10, 33]. It is also well established that NP cell apoptosis is a classical feature during disc degeneration and that inhibiting NP cell apoptosis is helpful to alleviate disc degeneration-associated pathology [34]. However, the molecular mechanisms of NPC apoptosis under high compressive stress remain unclear.

It has been widely reported that SIRT1 can repress the process of IDD via various pathways [5, 35, 36].The present study found that the level of SIRT1 was decreased but cell apoptosis was enhanced in human degenerative disc samples, which revealed a possible relationship between SIRT1 and IDD. Furthermore, SIRT1 overexpression induced by LV-SIRT1 dramatically reduced cell apoptosis in rat NPCs under high-magnitude compression in a 3D cell culture model. Several studies have reported that SIRT1 protects degenerative NPCs against apoptosis by activating autophagy [9, 12, 22]. Notably, our recent study also demonstrated that SIRT1 overexpression can effectively alleviate senescence in NPCs under high compressive stress by recycling injured mitochondria via mitophagy [23]. Accordingly, in the present study, we investigated whether SIRT1 attenuated high compression-induced apoptosis by regulating autophagy in vitro. As expected, SIRT1 overexpression strongly upregulated the expression of the autophagy marker LC3B but downregulated the expression of P62. Furthermore, both immunofluorescence and TEM analysis showed more autophagosomes in SIRT1-overexpressing NPCs in the 3D cell culture model under high-magnitude compression. Conversely, upregulation of SIRT1 considerably decreased the expression of Bax and cleaved caspase 3 but increased the expression of Bcl-2. In line with this, TUNEL staining and flow cytometry analyses of the 3D NPC culture model under high-magnitude compression also showed a lower NPC apoptosis ratio after SIRT1 overexpression. These results indicate that overexpression of SIRT1 inhibited NPC apoptosis under high-magnitude compression by regulating the autophagy process. To further verify this hypothesis, an in vivo rat tail compression model was constructed. Consistently, SIRT1 overexpression strengthened autophagy and attenuated apoptosis in this in vivo model, which contributed to suppression of IDD.

Emerging evidence suggests that the formation of the Fas/LC3B complex plays a crucial role in the interaction between autophagy and cell apoptosis in various disease models [15–17]. In the current study, we demonstrated that LC3B directly interacted with the apoptotic signaling molecule Fas under high-magnitude compression. SIRT1 overexpression obviously increased formation of the LC3B/Fas complex, which rapidly alleviated the activation of the NF-*κ*B pathway and thereby inhibited cleavage of caspase 3. In addition, we found that LC3B silencing alleviated the inhibition of the NF-*κ*B signaling pathway, thereby partially counteracting the cleavage of caspase 3 and inhibiting NPC apoptosis under high-magnitude compression. Previous convincing experimental data have demonstrated that engagement of Fas with FasL increases RelA/P65 phosphorylation, indicating NF-*κ*B activation [37, 38]. On the other hand, other compelling data have shown that NF-*κ*B enhances cleavage of caspase 3 to trigger apoptosis in NPCs [39, 40]. We can draw from these reports that the elevation in Fas consumption due to higher combination of LC3B and Fas leads to obstruction of NF-*κ*B activation and ultimately inhibition of cell apoptosis.

However, there are several limitations in this study. First, some studies have reported that Fas-LC3B binds to caveolin-1 under hyperoxia [23], and whether this phenomenon is true under high pressure stress needs further study. Second, dynamic compressive stress was used in the in vitro cell experiments, whereas static pressure was used in the animal model due to a lack of suitable experimental equipment. If possible, to resolve this limitation, we will develop a mechanical system that can apply various dynamic compression to individual discs. Third, the magnitude of the in vitro dynamic compression was 20% according to our previous experience [23], while the magnitude of the in vivo compression was only 10% because we found that a magnitude of 20% compression led to a series of adverse reactions (i.e., microfracture of vertebral bone, loosening of the Kirschner wires, and self-absorption of intervertebral discs). We deduce that this issue may be related to differences in the mechanical characteristic of the hydrogel and vertebral bone. Based on our continued exploration, we found that a magnitude of 10% compression was suitable for rat tail in vivo experiments. Fourth, because T2-weighted MRI is a common technique to observe intervertebral disc degeneration, we only used MRI scanning to compare disc changes among the four different experiment groups at the last time point. Although the changes in disc height can be reflected in part by MRI, obtaining an X-ray image at the initial and final stage to compare changes in disc height among the groups would significantly improve our study.

## 5. Conclusion

In the present study, a 3D cell culture model and in vivo rat tail compression model were constructed, and analyses of these models revealed that SIRT1 overexpression can increase formation of the LC3B/Fas complex, which contributes to suppression of NPC apoptosis under high-magnitude compression through inhibition of the NF-*κ*B pathway (Figure 7).

## Figures and Tables

**Figure 1:** High-magnitude compression aggravated cell apoptosis and attenuated SIRT1 expression in rat NPCs. (a) The main units of the substance exchanger-based perfusion bioreactor (1: substance exchanger; 2: medium reservoir; 3: tissue culture chambers and pressure stress application system; 4: peristaltic pump; 5: pH, PO_2_, and CO_2_ sensor). (b, c) The apoptosis rate and SIRT1, p-P65, and apoptosis-related protein (Bcl-2, Bax, and cleaved caspase 3) levels in NPCs exposed to different compressive deformations (0% and 20%) were examined by flow cytometry and western blotting, respectively. (d) The expression of SIRT1 in NPCs exposed to different compressive deformations (0% and 20%) was examined by immunofluorescence. ^∗^*P* < 0.05 vs. the 0% (control) compressive deformation group. White bars = 100 *μ*m. NPCs: nucleus pulposus cells.

**Figure 2:** Observation of SIRT1 expression, cell apoptosis, and autophagy in human-degenerated NP samples. (a) Representative lumbar MRI images showing grade I-II and grade V discs in LVF (left) and IDD (right), respectively. Red arrows indicate the target NP tissue. (b, c) Immunohistochemical staining and western blotting results showing the expression of SIRT1, LC3B, and cleaved caspase 3 in NP tissue from LVF and IDD patients. Black bars = 100 *μ*m. ^∗^*P* < 0.05 vs. the LVF group. NP: nucleus pulposus; LVF: lumbar vertebral fracture; IDD: intervertebral disc degeneration.

**Figure 3:** SIRT1 overexpression enhanced autophagy and reduced cell apoptosis in rat NPCs under high-magnitude compression. (a) The efficiency of SIRT1 overexpression was detected via quantitative real-time PCR and western blotting. (b) The expression levels of autophagic biomarkers (LC3B and P62) and apoptosis-related proteins (Bcl-2, Bax, and cleaved caspase 3) in each group were analyzed by western blotting. (c) Formation of autophagosomes detected by analyzing SQSTM1/P62 immunofluorescence in NPCs before and after SIRT1 overexpression under high-magnitude compression. (d) Autophagosomes in NPCs were examined via TEM. Red arrows show characteristic double-membrane autophagosome formation. (e, f) The apoptosis rate of the NPCs in each group was analyzed via flow cytometry and TUNEL staining. ^∗^*P* < 0.05 vs. the 0% (control) compressive deformation group. White bars = 100 *μ*m. Black bars = 1 *μ*m. NPCs: nucleus pulposus cells; PCR: polymerase chain reaction.

**Figure 4:** SIRT1 overexpression increased formation of the LC3B/Fas complex and inhibited activation of the NF-*κ*B pathway. (a) Immunoprecipitation assay results showing the amount of LC3B/Fas complex in SIRT1-overexpressing NPCs compared with control cells. Briefly, the cell lysates were immunoprecipitated (IP) with anti-FAS antibody, and the immunoprecipitated proteins were examined via western blotting using an anti-LC3B antibody. (b): Western blotting results showing the levels of P65 and p-P65 in NPCs with or without LV-SIRT1 exposed to high compressive stress. ^∗^*P* < 0.05 vs. the 0% (control) compressive deformation group. ^#^*P* < 0.05 vs. the 20% compressive deformation group. NPCs: nucleus pulposus cells.

**Figure 5:** Downregulation of LC3B alleviated the inhibition of the NF-*κ*B signaling pathway and aggravated apoptosis in SIRT1-overexpressing NPCs under high-magnitude compression. (a) The efficiency of LC3B-siRNA was examined via western blotting. (b) The levels of cleaved caspase 3, P65, and p-P65 in NPCs were detected by western blotting. (c, d) The apoptosis rate of NPCs was examined via flow cytometry and TUNEL staining. ^∗^*P* < 0.05 vs. the 20% compressive deformation group. ^#^*P* < 0.05 vs. the 20%+SIRT1 compressive deformation group. White bars = 100 *μ*m. NPCs: nucleus pulposus cells.

**Figure 6:** SIRT1 overexpression rescued autophagy and reduced cell apoptosis in a rat tail compression model. (a) Appearance and X-ray views of the modified rat tail static compression model. (b) T2-weighted MRI image of the experimental rat tail IVD under high-magnitude compression at 4 weeks in each group. (c) Histomorphological changes in the experimental rat tail IVD under high-magnitude compression. (d) Immunohistochemical staining of cleaved caspase 3, LC3B, and p-P65 expression in experimental rat tail IVD samples from each group. White bars = 500 *μ*m. Black bars = 100 *μ*m. ^∗^*P* < 0.05. ^#^*P* > 0.05. IVD: intervertebral disc; IDD: intervertebral disc degeneration.

**Figure 7:** Schematic diagram showing the potential mechanism by which SIRT1 upregulation modulates high-magnitude compression-induced NPC apoptosis in this study. NP cell apoptosis is a main cellular pathological feature during IDD, which ultimately contributes to aggravation of IDD. In this study, our result demonstrated that upregulation of SIRT1 expression increased formation of the LC3B/Fas complex, which contributed to suppression of NPC apoptosis under high-magnitude compression via inhibition of the NF-*κ*B pathway. IDD: intervertebral disc degeneration.

**Table 1:** Primers for target genes.

Gene	Primer sequence (5′-3′)
SIRT1	F: GCTCGCCTTGCTGTGGACTTC
	R: GTGACACAGAGATGGCTGGAACTG
*β*-Actin	F: CCGCGAGTACAACCTTCTTG
	R: TGACCCATACCCACCATCAC

## Data Availability

The data generated for this study are all included in the manuscript.
